The article "Congenital Cataract Surgery: A Retrospective Analysis of 62 Patients in a Developing Country" was retracted in 2023. Reasons: unreliable results or conclusions; lack of ethics approval or compliance; concerns about the data; concerns about the peer review.

# Congenital Cataract Surgery: A Retrospective Analysis of 62 Patients in a Developing Country

**DOI:** 10.1155/2021/6431276

**Published:** 2021-12-23

**Authors:** Raed Shatnawi, Motasem Al-Latayfeh, Mohammad Abu-Ain

**Affiliations:** ^1^Department of General and Special Surgery, Faculty of Medicine, The Hashemite University, Zarqa, Jordan; ^2^Department of Ophthalmology, Prince Hamza Hospital, Amman, Jordan

## Abstract

**Purpose:**

This study was aimed at describing our experience in congenital cataract surgery in a developing Country.

**Methods:**

A retrospective study was conducted in Amman, Jordan. The patients who were diagnosed with congenital cataract and underwent the surgery were included in the study. It was decided to use an intraocular lens if the corneal diameter was more than 10 millimeters.

**Results:**

The findings revealed that around 13 of the patients did not have any visual axis opacification, indicating that they were aphakic. Visual axis opacification was seen in 8 out of the total sample of participants. Eleven patients with obvious opacification of the visual axis were found to be pseudophakic after at least two procedures and were thus cleared. It was necessary to do a second surgery to rectify the visual axis opacification induced by pseudophakia, which was putting the patient's ability to recuperate at danger. Three of them (or 12 percent) exhibited visual axis opacification, which is a rare occurrence. The intraocular lenses used in the remaining 24 patients were constructed of hydrophilic plastic.

**Conclusion:**

Patients are less prone to have visual axis opacification while implanted by hydrophobic intraocular lenses is something they should consider.

## 1. Introduction

Possessing a congenital cataract in a kid has been associated with an elevated risk of juvenile blindness in studies conducted on this population [1–3]. When the natural lens of the eye becomes clouded with increasing age, this is referred to as a cataract. Congenital cataracts in newborns are common and may be caused by pharmaceutical reactions, inflammation, genetic diabetes, trauma, infection, susceptibility, or metabolic abnormalities [4, 5]. The use of tetracycline antibiotics during pregnancy to treat infection may result in the development of a congenital cataract as a side effect [2, 3].

In the case of congenital cataracts, issues emerge as a result of the creation of crucial proteins that are required to preserve the clarity of the native lens. Recently developed surgical techniques have had a substantial impact on the outcomes of cataract surgery in neonates, which has been shown to be significantly improved [4]. However, complications will always occur, whether during surgery, soon thereafter, or in the years that follow [2, 4].

The article "Congenital Cataract Surgery: A Retrospective Analysis of 62 Patients in a Developing Country" was retracted in 2023. Reasons: unreliable results or conclusions; lack of ethics approval or compliance; concerns about the data; concerns about the peer review.

The most common complication of intraocular lens (IOL) implantation is secondary opacification of the visual axis, which occurs most often in newborns and is caused by cortical reproliferation. This is the most common complication of this procedure [6–8]. The use of an IOL may result in IOL degradation, inflammation, secondary membranes, and the need for further surgeries, all of which are undesirable outcomes. In certain cases, surgeons may be able to avert poor outcomes by being aware of potential anomalies that are specific to infant eyes. It might help surgeons make more precise diagnoses and treat their patients more effectively [6, 9, 10].

Congenital cataracts have posed a significant challenge to the treatment of curable childhood blindness throughout the past few decades [1, 2]. Although age is the most major risk factor for congenital cataract, there are many other factors to consider. When it comes to congenital cataract surgery, the posterior capsule management, robust amblyopia therapy, and refractive management all have a part in the outcome of the procedure [1, 2, 11].

A variety of surgical techniques have been developed to reduce the incidence of posterior capsular opacification. The surgical therapy for congenital cataracts is posterior chamber IOL implantation with anterior vitrectomy and posterior capsulotomy, which is usually acknowledged as the gold standard [4, 7]. It is controversial whether or not an anterior vitrectomy and posterior capsulotomy should be performed at a certain age or not. Compared to established regions, the prevalence of this illness has grown tenfold in emerging areas, with 1-15 children out of every thousand suffering from it in developing countries. Despite its poor visual outcomes, pediatric cataract surgery is still the primary therapeutic option [4, 7].

Cataract surgery in children may have severe intraoperative and postoperative implications for children with a variety of medical conditions. Postoperative complications may include nystagmus and other vision problems such as glaucoma and strabismus. Due to a lack of equipment, money, methods, and health ministry strategic plans, effective and prompt treatment is also limited to developed areas [7, 8, 11–13].

Congenital cataract surgery is a demanding procedure that requires the use of advanced technology and close attention to detail. Congenital cataract surgery is fraught with controversy because of disagreements about the appropriate time and method to use. It is critical to have population-based information on surgical care and to conduct epidemiological research in order to improve management and preventative measures, particularly in developing nations [1, 2, 11].

The article "Congenital Cataract Surgery: A Retrospective Analysis of 62 Patients in a Developing Country" was retracted in 2023. Reasons: unreliable results or conclusions; lack of ethics approval or compliance; concerns about the data; concerns about the peer review.

The Prince Hamza Hospital in Amman, Jordan, is the only pediatric ophthalmology referral hospital in the nation and the largest in the Middle East. It was founded in 1982. Data on the incidence and frequency of congenital cataracts in Jordan, on the other hand, are few in published research. Given that an infant's eye responds differently than an adult's eye, congenital cataract surgery should only be performed in institutions that are appropriately equipped to manage the complicated treatment. In order to get the greatest possible vision and limit the risk of acquiring glaucoma later on in life, congenital cataract surgery should be performed as soon as feasible after the patient's birth.

Delaying cataract surgery may have significant repercussions for a person's ability to see well. Babies born with congenital cataracts have a decreased chance of regaining their vision if the cataract is not removed within the first few months of life. Consequently, the major objective of the research was to discuss our experience with congenital cataract surgery in a poor country. Furthermore, the various factors that impact anatomical and functional results following surgery for a congenital cataract were investigated in this study.

## 2. Materials and Methods

The patients in this retrospective study were those who had been diagnosed with congenital cataract and had been operated on by the surgeon at Prince Hamza Hospital at the time of their diagnosis. All of these patients were seen by the same surgeon, who treated them all. In situations where the corneal diameter was more than 10 mm, an intraocular lens (IOL) was implanted that was about the same size as the diameter of the capsular bag, resulting in a clear vision. There has been a decision to employ intraocular lenses (IOLs) since they provide partial correction whereas other optical devices, such as contact lenses and aphakic glasses, need a larger degree of conformity. It was decided to enroll infants who had thick opacity over the whole lens and were older than 37 weeks of gestation as participants in the study.

Individuals with persistent primary hyperplastic vitreous, ocular injuries, corneal problems, glaucoma, a history of Lower syndrome, or rubella, on the other hand, were excluded from the research. Either they were congenital, which means that they were there from birth, or they might have developed as a result of a trauma such as a car accident, according to the findings of the research. It was also agreed that patients who did not finish the follow-up and who did not have normal pupil dilation would be ruled out of consideration for future research. Before taking part in the research, all of the patients who were included in it were asked to sign an informed written permission form, which they did.

The article "Congenital Cataract Surgery: A Retrospective Analysis of 62 Patients in a Developing Country" was retracted in 2023. Reasons: unreliable results or conclusions; lack of ethics approval or compliance; concerns about the data; concerns about the peer review.

Following the findings of this investigation, it was determined that the Prince Hamza Hospital is the only hospital in Jordan that delivers congenital cataract services under contract with the Ministry of Health.

Children who took part in the research ranged in age from babies to eight-year-olds, with the youngest being eight months old. A PPC, an anterior vitrectomy, and an intraocular lens implant were among the treatments performed as part of their limbal surgery, which also included additional procedures (in the bag). Following surgery, the patients were given dexamethasone intracameral injections as well as gentamicin/dexamethasone subconjunctival injections in each of the four quadrants of their eyes. Information from patients' medical records, such as their age at the time of surgery, whether or not they had intraocular lenses implanted, how many surgeries they had, what sort of therapy they received, and whether or not they had any complications, was evaluated.

The use of hydrophilic or hydrophobic acrylic IOLs as biocompatibility materials was made possible by the lengthy history of the material in clinical practice and its safety for intraocular implantation. The study identified which kind of intraocular lens (hydrophobic acrylic IOL or hydrophilic acrylic IOL) was used in the patient and then compared the effects of the two different therapies.

## 3. Results

As shown in Table 1, there were 62 people with congenital or developmental cataracts who were investigated, with 32 males and 30 females participating. After surgery on infants under the age of one year, seven patients were left aphakic and 10 were left pseudophakic.

Secondary membranes or an aberrant inflammatory response was not seen in any of the participants in the aphakic group. It was necessary to do a second procedure on two of the pseudophakic people to eliminate the obstruction in their visual axis. Pseudophakia afflicted 49 children, 25 of whom received a hydrophobic intraocular lens and 24 of whom had a hydrophilic IOL. There were three patients who developed VAO, which indicated the necessity for a second surgery in 33% of hydrophobic patients.

It was found that eight hydrophilic patients (33 percent) developed VAO and needed a second surgery. This was removed from one patient in the hydrophilic group after three procedures, and IOL explantation was performed. One-third of the group (13 patients) was aphakic, and none of the patients had VAO. Eleven of the 49 pseudophakic patients needed two or more procedures to remove the VAO, which represents a large proportion of the population. Twenty-five pseudophakic patients were fitted with hydrophobic intraocular lenses, and three (12 percent) of them developed VAO.

The article "Congenital Cataract Surgery: A Retrospective Analysis of 62 Patients in a Developing Country" was retracted in 2023. Reasons: unreliable results or conclusions; lack of ethics approval or compliance; concerns about the data; concerns about the peer review.

There were 24 patients in all, with 8 (33 percent) developing VAO, suggesting the need for a second procedure. Following the initial IOL, these eight patients received hydrophilic IOLs. In the course of the study, 22 patients were lost to follow-up; however, those who remained were investigated, and it was discovered that 8 of them were aphakic or pseudophakic in nature. 17 patients (27 percent) were found to be lost, with seven of those patients being aphakic. One of the patients had microphthalmia, while the other had a high intraocular pressure (IOP) before the cataract surgery. Both were treated successfully.

Atypical inflammatory reactions or secondary membranes were not seen in any of the patients who participated in the study. Pseudophakia patients were treated with hydrophobic intraocular lenses in six instances and hydrophilic intraocular lenses in the other four cases. VAO has not been experienced by anybody in the aphakic group. In the pseudophakic group, VAO was found in just two patients out of every 10 patients. According to the findings of the study, the risk of VAO is decreased when using a hydrophobic IOL. Thirteen of the patients studied were aphakic, which means that they did not have visual axis opacification in their visual field. 49 patients were found to be pseudophakic, and 22 percent of them had severe VAO, requiring two or more procedures to clear the visual axis, delaying the start of their visual rehabilitation.

Aphakic spectacles and contact lenses were used to visually rectify the condition of aphakia. They had to go through a period of visual rehabilitation once the procedure was completed. With the exception of endophthalmitis (1 case), dropped intraocular lenses (1 case), decentration (4 occurrences), and retinal detachment (in 1 patient, who was lost from F/U for 3 years due to a severe deep inflammatory reaction), the VAO-related issues found were the most prevalent. Among individuals who underwent cataract surgery, the researchers found no indication of glaucoma developing as a severe consequence. Some persons with bilateral cataracts vanished for two or three years after having an F/U procedure performed on one eye. They then reappeared.

## 4. Discussion

As a consequence of technical improvements, surgical procedures for congenital cataract surgery have advanced significantly in recent decades. Jordan's Ministry of Health facilities are home to just one pediatric ophthalmology service, which is situated at Prince Hamza Hospital in the country's capital, Amman, and serves children from birth to age 18.

The article "Congenital Cataract Surgery: A Retrospective Analysis of 62 Patients in a Developing Country" was retracted in 2023. Reasons: unreliable results or conclusions; lack of ethics approval or compliance; concerns about the data; concerns about the peer review.

Early surgical intervention in microophthalmic eyes is associated with an acceptable incidence of postoperative complications, in addition to excellent visual results [8]. Findings from previous studies have shown that congenital cataracts are linked and that this is an important basis for treating and preventing childhood blindness [2, 3, 8].

Improved microsurgical techniques, improved lens technology, and a better knowledge of refractive eye development have all contributed to the increased use of intraocular lenses in patients. The surgical method averted the development of the inflammatory membrane or posterior capsular opacification, resulting in a clean axis for the foreseeable future. Anesthesia was administered with the use of the proper equipment. We removed the posterior capsule with the use of a vitrectomy instrument. Following the results of recently completed clinical and laboratory tests, it has been determined that treatment protocols must be modified in order to give children with a decent binocular visual experience throughout their early years of life [2, 4].

Additional factors that may have an impact on stereoacuity outcomes include the length of the operation, the severity of the postsurgical consequences, the treatment regimen, and the method used to test stereoacuity [4, 8]. When the patients had cataract surgery to remove the growing cataracts, their binocular vision improved both at a distance and in the near field of vision.

Despite this, strabismus and myopia were seen in a lower proportion of the individuals. According to the research's postsurgical data, growing cataracts showed improved functional results when compared to congenital cataracts in the studied population. Drug exposure during pregnancy, ionizing radiation exposure during pregnancy, and gestational diabetes mellitus have all been linked to cataract development [1–3, 9].

Despite the fact that glaucoma was not shown to be a serious issue in this study, one of the patients with bilateral cataracts was lost from the study following treatment in one eye, only to reappear 2 or 3 years after the first treatment [2, 3]. Glaucoma was not shown to be a significant problem in this research; nevertheless, one of the patients with bilateral cataracts was lost from F/U after treating one eye, only to resurface 2 or 3 years later.

Visual loss caused by congenital cataracts causes dislocation of binocular cortex development during the acute period, resulting in impaired stereoacuity in the majority of cases [2]. Lens formation occurs via DNA-binding transcription factors, which are especially abundant in the lens. They also discussed current techniques and assistance for human pediatric cataracts in clinical research as well as human genetic studies [1, 4].

The article "Congenital Cataract Surgery: A Retrospective Analysis of 62 Patients in a Developing Country" was retracted in 2023. Reasons: unreliable results or conclusions; lack of ethics approval or compliance; concerns about the data; concerns about the peer review.

The discoveries have assisted in the identification of original cataract-associated genes, which will aid in the development of a comprehensive understanding of the genetic basis of these abnormalities and remedies. A problematic aspect of congenital cataract surgery is the need for specialized tools, as well as a lengthy recuperation time after the procedure is completed [7, 8]. Primary intraocular lens implantation increased best-corrected visual acuity in microphthalmic eyes following congenital cataract surgery in the absence of cataract [1, 6].

There were also few or no postoperative complications in the cases presented, suggesting that there were no intraoperative issues. Primary intraocular lens (IOL) implantation may be performed within the first year of life if the necessary safeguards are taken. Previous research findings support the results reached in this study [1, 6, 10].

Contrast sensitivity, stereopsis, and visual acuity were all shown to have an influence on patient satisfaction with their quality of life after cataract surgery, according to a recent study. The present inquiry is conducted in a similar way. It was advised to participants with infant aphakia who were enrolled in the Infant Aphasia Therapy Trial that they should not have a secondary intraocular lens placed for at least five years before [1, 2].

Three patients under the age of five years had their intraocular lenses (IOLs) swapped because they had developed myopic refractive defects as a consequence of the axial length of the eye becoming longer. Neither the aphakic nor the pseudophakic groups showed statistically significant differences in visual outcomes.

## 5. Conclusion

In the present study, a number of factors impacting morphological and functional outcomes after surgery for a congenital cataract were investigated. The results revealed that it is vital that bilateral surgery be promoted in poor countries in order to track down patients who have not shown up for further follow-up appointments. Pseudophakia was shown to be responsible for a higher percentage of patients not being followed up. As a result of the fact that it is a retrospective study, the information acquired is neither complete nor accurate. The research has a number of flaws, which are significant. As a consequence of scarcity of accurate data, the visual outcomes of cataract surgery were not included in the study. The study was a success despite its limitations since it brought attention to an important public health issue impacting the Jordanian people and one that has a direct impact on surgical results. Patients who had gone through the holes in the follow-up procedure had previously been identified as having a need for a service, according to the results of the investigation. When done successfully, bilateral surgery should be encouraged in the same operation.

The article "Congenital Cataract Surgery: A Retrospective Analysis of 62 Patients in a Developing Country" was retracted in 2023. Reasons: unreliable results or conclusions; lack of ethics approval or compliance; concerns about the data; concerns about the peer review.

## Figures and Tables

**Table 1:** Characteristics.

Characteristics	*N* (%)
Males	32 (52%)
Females	30 (48%)
Bilateral	41 (66%)
Unilateral	21 (34%)
Less than 1 year	17 (27%)
Aphakic	13 (21%)
Pseudophakic	49 (79%)
Hydrophobic IOL	49 (79%)
Hydrophilic IOL	24 (49%)

## Data Availability

All data used to support the findings of this study are included within the article.
